# Effects of Acupuncture and Moxibustion Combined with Needle-Knife on Pain and Lumbar Function in Patients with Lumbar Disc Herniation

This article has been retracted.

**DOI:** 10.1155/2022/9185384

**Published:** 2022-04-07

**Authors:** Guoqiang Peng, Yanfang Zheng, Dejun Luo

**Affiliations:** ^1^Orthopedics Department of Traditional Chinese Medicine, Taizhou Jiangyan Hospital of Traditional Chinese Medicine, Taizhou, China; ^2^Comprehensive Nursing Clinic, PLA Rocket Force Characteristic Medical Center, Beijing, China; ^3^Department of Orthopedics, the People's Hospital of Jianyang City, Jianyang, China

## Abstract

This study aimed for the analysis of the effect of acupuncture and moxibustion combined with needle-knife on pain and lumbar function in patients with lumbar disc herniation. From June 2019 to February 2021, the medical records of 126 patients with lumbar disc herniation admitted to the department of orthopedics of our hospital were selected and divided into the control group (*n* = 63) treated with acupuncture and moxibustion and the observation group (*n* = 63) treated with acupuncture and moxibustion combined with needle-knife according to different treatment regimens. After 4 weeks of treatment, the clinical efficacy, pain status, and lumbar function were compared between the two groups. The concentrations of relevant inflammatory factors (IL-6, IL-10, TNF-*α*, and MMP-2) in peripheral blood of the two patients before and after treatment were measured by enzyme-linked immunosorbent assay (ELISA). After treatment, the overall response rate was 93.65% in the observation group, which was higher than 80.95% in the control group (*P* < 0.05); the visual blurred score (VAS) scores of lower limbs and waist in the observation group were lower than those in the control group, while the expression of pain mediators serotonin (5-HT) and prostaglandin E2 (PEG2) was also lower than that in the control group (*P* < 0.05); the Oswestry disability index (ODI) in the observation group was lower than that in the control group, while the Japanese Orthopedic Association assessment treatment score (JOA) was higher than that in the control group (*P* < 0.05). After treatment, the concentration levels in peripheral blood (IL-6, IL-10, TNF-*α*, and MMP-2) were significantly lower in the observation group than in the control group (*P* < 0.05). Acupuncture and moxibustion combined with needle-knife is effective in the treatment of lumbar disc herniation, which helps to improve the clinical efficacy, relieve pain symptoms, promote the improvement of lumbar function, and contribute to the reduction of inflammatory factors.

## 1. Introduction

Lumbar disc herniation is a very common clinical disease in orthopedics, that is, disc degeneration, herniated nucleus pulposus, and annulus fibrosus rupture cause stimulation and compression of cauda equina and nerve roots, resulting in disease syndrome, mostly caused by dysplasia, disc degeneration, genetics, and other factors, which is one of the main factors leading to back and leg pain [1, 2].

Western surgery is a common clinical treatment for lumbar disc herniation, but it is highly invasive and prone to recurrence after surgery, and its application is controversial [3]. With the further study of Chinese medicine, Chinese medicine has been applied to patients with lumbar disc herniation, and the common solutions are acupoint application, acupuncture and moxibustion, and oral Chinese medicine. Among them, acupuncture and moxibustion are pure green treatment solutions, and their advantageous diseases are painful diseases, of which lumbar disc herniation is one type, which can effectively relieve patients' painful symptoms in the back and legs [4]. However, if a patient with lumbar disc herniation has positive symptoms of abdominal pressure pain or a significantly smaller lumbar curve, local treatment with acupuncture is slow to take effect, and the effectiveness of single treatment needs to be improved [5].

Needle-knife is a new type of minimally invasive surgical solution based on the concept of combined Chinese and Western medicine treatment, with the advantages of low price, convenient operation, and significant effect. Lumbar disc herniation belongs to the advantages of this treatment and meets its indications. Through needle-knife treatment, the soft tissue in the spinal canal can be restored to dynamic balance, so as to achieve the therapeutic goal [6].

The purpose of this study is to analyze the effect of acupuncture and moxibustion combined with needle-knife on the improvement of pain and lumbar function in patients with lumbar disc herniation and to evaluate the clinical efficacy, pain status, lumbar function, and associated inflammatory factor level changes as indicators.

## 2. Materials and Methods

### 2.1. Basic Information

This study included 126 patients with lumbar disc herniation, including 63 cases in the control group and 63 cases in the observation group. The basic information was no significant difference in the general data between the two groups (*P* > 0.05), as given in Table 1.

### 2.2. Inclusion and Exclusion Criteria

The inclusion criteria were as follows: the condition was consistent with the relevant criteria in the Chinese Expert Consensus on Pain in the Diagnosis and Treatment of Lumbar Disc Herniation [7], and the diagnosis was confirmed after diagnosis; the age ranged from 18 to 75 years; there were symptoms of abdominal muscle tenderness and smaller lumbar curvature; acupuncture and needle-knife treatment were performed for the first time; the cognitive ability, comprehension ability, communication ability, and language communication ability were normal; and the compliance was good. Exclusion criteria were as follows: low back pain due to other diseases; patients combined with lumbar disc herniation calcification, radiculitis, spinal stenosis, and lumbar tuberculosis; patients with pregnancy or lactation; patients with mental disorders or malignant tumors; and patients combined with severe organ dysfunction.

### 2.3. Methods

The study protocol was approved by Taizhou Jiangyan Hospital Ethics Committee. The medical records showed that all patients received all-round examination, and 63 patients were treated with acupuncture and moxibustion, that is, after locating the responsible intervertebral space, Weizhong, Huanqiao, Yaojiaji, and Yanglingquan points were selected, and acupuncture was given by vertical needle insertion. The needle could be inserted 1–2.5 inches. After determining deqi, the needle was retained for 30 minutes, and acupuncture was performed every 2 days for 4 weeks. The above patients were retrospectively divided into the control group. The other 63 cases were treated with acupuncture and moxibustion combined with needle-knife, in which the acupuncture therapy was the same as the control group. During needle-knife treatment, the prone position was taken, and the painful nodular points 0.5 cm, 1.5 cm, and 3-4 cm beside the spinous process were located by gentian violet. After local anesthesia, the needle-knife was inserted about 4-5 cm, and deep fasciolysis was performed. The upper and lower painful tubercle points of the iliac wing were repositioned, about 1-2 cm of the needle-knife was inserted, and superficial fascia release was performed. Through the course of the sciatic nerve, three painful nodular points were selected to penetrate 1-2 cm into the needle-knife and released with superficial fascia. Needle-knife treatment was performed once or twice a week for 4 weeks. The above patients were retrospectively divided into the observation group.

### 2.4. Observation Index

(1) The efficacy of the treatment was assessed based on the improvement of the Japanese Orthopedic Association assessment treatment score (JOA), combined with clinical performance. If the pain in the lower back and leg has disappeared, the range of movement has increased, the sensory function and muscle strength of the affected limb have returned to normal, the straight leg raise can be ≥70°, the ability to perform daily activities has basically returned, and the improvement rate of JOA score is 90% or more, then the patient is clinically cured; if the pain in the lower back and leg is significantly relieved, the ability to perform activities has improved, the pain in the lower limb and numbness in the lower limb occur under exertion, and the improvement rate of JOA score is 60%–89%, then the patient is clinically cured. If the pain in the lower back and legs is relieved and the improvement rate of JOA score is 30–59%, it is effective; if the pain in the lower back and legs is not changed or even aggravated, the ability of daily activities is limited, and the improvement rate of JOA score is <30%, it is not effective [8]. (2) Pain status: the pain condition of the lower limbs and low back was assessed by visual ambiguity scoring (VAS) before and after the treatment in both groups, and the pain condition was marked on a scale of “0–10,” with 0 being no pain and 10 being severe pain [9]. At the same time, a 3 ml elbow vein blood sample was centrifuged at 3000 r/min × 10 min, and the supernatant was extracted for the determination of pain mediators 5-hydroxytryptamine (5-HT) and prostaglandin E2 (PEG2) expression by enzyme-linked immunosorbent assay. (3) Lumbar spine function: the Oswestry dysfunction index (ODI) and JOA scores were used to assess lumbar spine function before and after treatment in both groups. The ODI contains 10 scoring items with a total score of 100, the higher the score obtained, the greater the degree of dysfunction [10]; the JOA contains 4 dimensions with a total score of 29; the higher the score obtained, the better the level of function [8]. (4) Peripheral blood was collected from patients in both groups before and after completion of the treatment course, and the serum was isolated and frozen for further use. The relative inflammatory cytokines IL-6, IL-10, TNF-*α*, and MMP-2 concentration levels were measured in peripheral blood of the two patients before and after treatment according to the method of ELISA kits.

### 2.5. Statistical Analysis

Statistical Product and Service Solutions (SPSS) statistical software (version 25.0) (IBM, Armonk, NY, USA) was used for comparative analysis of the study indicators. The comparison of counting data was performed by the *χ*2 test, represented by (*n* (%)); the comparison of measurement data were performed by the *t*-test, represented by (‾*x* ± *s*). *P* < 0.05 indicates a significant difference between groups.

## 3. Results

### 3.1. Comparison of the Clinical Outcomes of the Two Groups of Patients

In terms of clinical efficacy, 13 cases were clinically cured, 26 cases were significantly effective, 20 cases were effective, and 4 cases were ineffective, with an overall response rate of 93.65%; in the control group, 7 cases were clinically cured, 18 cases were significantly effective, 26 cases were effective, and 12 cases were ineffective, with an overall response rate of 80.95%, and the observation response rate was higher than that in the control group (*X*^2^ value = 4.582, *P*=0.032), as given in Table 2.

### 3.2. Comparison of Pain Status between the Two Groups

In terms of pain status, there was no significant difference in VAS score and 5-HT and PEG2 expression in lower limbs and waist before treatment between the two groups (*P* > 0.05). After the course of treatment, the pain status of the two groups was improved, VAS score, 5-HT, and PEG2 expression in lower limbs and waist were decreased, and the observation group was lower than the control group (*P* < 0.05), as given in Table 3.

### 3.3. Comparison of Lumbar Function between the Two Groups

In terms of lumbar function, there was no significant difference in ODI and JOA scores before treatment between the two groups (*P* > 0.05). After the course of treatment, the lumbar function of the two groups was improved, and the ODI score of the observation group was lower than that of the control group, while the JOA score was higher than that of the control group (*P* < 0.05), as given in Table 4.

### 3.4. Comparison of Inflammatory Factors between the Two Groups

Before treatment, there were no significant differences in the levels of IL-6, IL-10, TNF-*α*, and MMP-2 in peripheral blood between the control group and observation group (*P* > 0.05). After each treatment, the concentrations of IL-6, IL-10, TNF-*α*, and MMP-2 in peripheral blood of patients in the observation group were significantly lower than those in the control group (*P* < 0.05), as shown in Figures 1–4.

## 4. Discussion

Lumbar disc herniation is mainly manifested as decreased lumbar range of motion, lumbar pain, scoliosis, and sciatica. In recent years, the incidence rate has been increasing year by year and shows a tendency of rejuvenation. It has become one of the common diseases affecting human health [11]. Cosamalón-Gan et al. [12] found that there is a close relationship between the generation of lumbar disc herniation and inflammatory response and mechanical compression; the pulp nucleus in the herniated disc compresses the nearby healthy tissue, resulting in an ischemic state of the nerve root, in addition to annulus fibrosus rupture causing chemical irritation, causing an immune response and aggravating the degree of nerve root inflammation. Moreover, the protrusion produces traction and compression effects on the nerve roots, resulting in blockage of local venous blood return, aggravating the degree of nerve root edema, impaired lumbar function, and increased sensitivity to pain, so when treating, attention should be paid to the relief of the degree of pain and improving its lumbar function [13].

According to the symptoms of lumbar disc herniation, it is attributed to the category of lumbar paralysis in traditional Chinese medicine. The causes of the disease are kidney Qi deficiency and muscle and bone stasis, mostly due to the invasion of cold and dampness evil and the flashing of falling servants, resulting in qi and blood disharmony and meridian obstruction, no general pain, which causes the disease and requires promoting blood circulation to remove blood stasis, dispersing cold and dredging wind, and dredging collaterals to relieve pain [14].

The main clinical treatment of lumbar disc herniation is conservative treatment and surgical treatment, acupuncture is one of the common conservative therapies, but Zai et al. [15] found that acupuncture alone in the treatment of lumbar disc herniation for relieving the degree of low back pain in patients and improving the degree of lumbar dysfunction remains to be improved. Needle-knife therapy is based on the meridian theory of traditional Chinese medicine, synthesizing the characteristics and advantages of needle and knife, using needle manipulation and meridian stimulation, through longitudinal and transverse dredging and dissection, release adhesive tissue, and promote the improvement of local microcirculatory function. Wang et al. [16] found through animal experiments that needle-knife therapy relieves local pain sensation and promotes improved mechanical properties of quadriceps tendon traction in rabbits with knee osteoarthritis.

In this study, the overall response rate after treatment in the observation group was higher than that in the control group, the VAS score of lower limbs and waist was lower than that in the control group, and the expression of 5-HT and PEG2 was also lower than that in the control group (*P* < 0.05), suggesting that the observation of acupuncture combined with needle-knife treatment was superior to the control group of acupuncture alone in improving the efficacy and relieving pain, which was consistent with the study results of Yang et al. [17]. Both 5-HT and PEG2 are common clinical pain mediators, and 5-HT is widely distributed in the central nervous system and peripheral tissues and is involved in pain regulation; PEG2 is a common mediator transmitting pain that can activate nociceptors, promote the massive release of *β*-endcurry peptide, and exacerbate the degree of pain [18].

Acupuncture and moxibustion combined with needle-knife regimen was used to treat patients with lumbar disc herniation. In acupuncture therapy, acupuncture was performed at Weizhong, Huanqiao, Yaojiaji, and Yanglingquan points to promote local blood circulation, exert the effects of soothing meridians and dispersing cold and relieving pain and dredging collaterals, achieve the effect of pain, dilate blood vessels, accelerate body metabolism, promote the timely absorption and dissipation of inflammatory factors, improve the degree of nerve root edema, effectively repair nerve roots, and relieve pain symptoms caused by compression of nerve roots.

Needle-knife therapy can effectively release adhesions, timely improve local microcirculatory function, stimulate the local peripheral nervous system, and reduce pain nerve sensitivity. The combination of the two therapies provides a synergistic effect, enhances efficacy, further mitigates the degree of aseptic inflammatory, promotes the timely resolution of inflammatory factor metabolites, and inhibits the production of pain mediators, thereby reducing VAS scores and 5-HT, PEG2 expression in the lower limbs and waist. In addition, in this study, the ODI score of the observation group after treatment was lower than that of the control group, while the JOA score was higher than that of the control group (*P* < 0.05), suggesting that the observation of acupuncture combined with needle-knife treatment is superior to the control group of acupuncture alone in promoting the improvement of lumbar function. Weizhong point belongs to the foot temple point; acupuncture and moxibustion deqi can promote the whole body Yang Qi smooth; Huanqiao point is in the sciatic nerve; acupuncture can make tendons and collaterals smooth; acupuncture at lumbar Jiaji point can promote blood circulation and remove blood stasis; Yanglingquan point can meridian antispasmodic. On the basis of acupuncture and moxibustion, needle-knife therapy was combined to release the tissue adhesion at the lesion site, relieve disc pressure, promote the timely relief of muscle spasm symptoms, improve the blood circulation at the lesion site, improve the degree of low back pain, and promote the effective recovery of lumbar function. Most studies have found that disc herniation can produce inflammatory factors, such as IL-6 and IL-10, which can stimulate nerve roots and cause pain or numbness [19, 20].

In this study, it was found that the levels of inflammatory factors IL-6, IL-10, TNF-*α*, and MMP-2 in peripheral blood of patients in the observation group were decreased more significantly after acupuncture and acupotomy treatment, indicating that acupuncture and acupotomy combined with acupotomy treatment can help reduce inflammatory factors in patients with lumbar disc herniation. The number of study cases was small, the observation time was short, the long-term efficacy and follow-up of patients were not statistically analyzed, and the indicators were subjective. In the later study, it is necessary to prolong the collection time of cases, expand the collection range, increase indicators, and make a multicenter study, so as to enhance the persuasion of study results.

## 5. Conclusion

Acupuncture and moxibustion combined with needle-knife are effective in the treatment of lumbar disc herniation, which helps to improve the clinical efficacy, relieve pain symptoms, and promote the improvement of lumbar function.

## Figures and Tables

**Figure 1:** The changes of IL-6 concentrations changes in peripheral blood detected by ELISA in two groups before and after treatment (x̅ ± *s*). ^*∗*^*P* < 0.05, compared with the control group.

**Figure 2:** The changes of IL-10 concentrations changes in peripheral blood detected by ELISA in two groups before and after treatment (x̅ ± *s*). ^*∗*^*P* < 0.05, compared with the control group.

**Figure 3:** The changes of TNF-*α* concentrations changes in peripheral blood detected by ELISA in two groups before and after treatment (x̅ ± *s*). ^*∗*^*P* < 0.05, compared with the control group.

**Figure 4:** The changes of MMP-2 concentrations changes in peripheral blood detected by ELISA in two groups before and after treatment (x̅ ± *s*). ^*∗*^*P* < 0.05, compared with the control group.

**Table 1:** Comparison of general information between the two groups.

Group	*n*	Gender (male/female)	Age (year)	Protruding segment			Course of disease (year)
				L_3-4_	L_4-5_	L_5-_S_1_	
Control group	63	33/30	52.71 ± 5.96	12	30	21	3.19 ± 0.33
Observation group	63	35/28	52.93 ± 6.01	13	31	19	3.22 ± 0.30
*X* ^2^/*t*	—	0.128	0.206	0.156			0.534
*P*	—	0.721	0.837	0.925			0.594

**Table 2:** Comparison of clinical efficacy between the two groups (*n* (%)).

Group	*n*	Clinical efficacy				Total effective rate
		Clinical cure	Markedly effective	Efficient	Invalid	
Control group	63	7 (11.11)	18 (28.57)	26 (41.27)	12 (19.05)	51 (80.95)
Observation group	63	13 (20.63)	26 (41.27)	20 (31.75)	4 (6.35)	59 (93.65)
*X* ^2^	—	—	—	—	—	4.582
*P*	—	—	—	—	—	0.032

**Table 3:** Comparison of pain status between the two groups (x̅±*s*).

Group (*n*)	Lower limb pain score (score)		Waist pain score (score)		5-HT level (*μ*mol/L)		PEG_2_ level (*μ*g/L)	
	Before therapy	After treatment	Before therapy	After treatment	Before therapy	After treatment	Before therapy	After treatment
Control group (*n* = 63)	6.59 ± 0.93	2.37 ± 0.33^a^	6.50 ± 0.39	2.61 ± 0.42^a^	1.00 ± 0.16	0.51 ± 0.11^a^	35.41 ± 6.03	25.77 ± 3.81^a^
Observation group (*n* = 63)	6.60 ± 0.90	1.70 ± 0.31^a^	6.47 ± 0.45	1.96 ± 0.31^a^	0.99 ± 0.18	0.31 ± 0.06^a^	35.45 ± 6.01	18.91 ± 3.30^a^
*t*	0.061	11.745	0.400	9.883	0.330	12.669	0.037	10.803
*P*	0.951	<0.001	0.690	<0.001	0.742	<0.001	0.970	<0.001

^a^Compared with the same group before treatment, *P* < 0.05.

**Table 4:** Comparison of lumbar function between the two groups (x̅±*s*, score).

Group (*n*)	ODI score		JOA score	
	Before therapy	After treatment	Before therapy	After treatment
Control group (*n* = 63)	45.45 ± 5.76	24.66 ± 4.17^a^	8.01 ± 2.16	16.88 ± 3.76^a^
Observation group (*n* = 63)	44.50 ± 5.70	17.03 ± 3.75^a^	8.00 ± 2.19	22.57 ± 3.03^a^
*t*	0.049	10.799	0.026	9.353
*P*	0.961	<0.001	0.979	<0.001

^a^Compared with the same group before treatment, *P* < 0.05.

## Data Availability

The datasets used and analyzed during the current study are available from the corresponding author upon request.
